This article has been retracted.

# Systematic Evaluation of Randomized Clinical Trials of Huangqin Tang in Combination with Mesalazine for Ulcerative Colitis

**DOI:** 10.1155/2022/2175913

**Published:** 2022-08-11

**Authors:** Chengyu Pan, Mengru Liu, Hui Li, Lanfu Wei, Pengcheng Wang, Kexuan Wu, Xing Ji, Limei Gu, Yaozhou Tian

**Affiliations:** ^1^Affiliated Hospital of Integrated Traditional Chinese and Western Medicine, Nanjing University of Chinese Medicine, Nanjing, Jiangsu 210028, China; ^2^Jiangsu Province Academy of Traditional Chinese Medicine, Nanjing, Jiangsu 210028, China; ^3^Community Health Service Center of Haicheng, Jianye, Nanjing, Jiangsu 210000, China; ^4^, Children's Hospital of Nanjing Medical University, Nanjing, Jiangsu 210028, China

## Abstract

**Objective:**

To systematically evaluate the efficacy and safety of Huangqin Tang (HQT) combined with mesalazine for the treatment of ulcerative colitis (UC).

**Methods:**

The China Knowledge Network, Wanfang Data, VIP, PubMed, SinoMed, Embase, and Cochrane Library databases were searched for randomized controlled trials (RCTs) of UC with HQT in Chinese and English. The search time was from the establishment of the database to October 2021. The included literature was evaluated for data extraction and risk of bias, efficacy and safety were evaluated using the RevMan5.3 software, and the quality of evidence was evaluated using GRADE.

**Results:**

Six studies with a total of 565 subjects were included, and a meta-analysis showed that HQT combined with mesalazine for UC significantly improved the cure rate (RR = 1.56, 95% CI [1.23, 1.98), *P*=0.0003) and overall efficacy rate (RR = 1.24, 95% CI [1.14, 1.35], *P*=0.00001), which significantly reduced the clinical symptom scores; however, all had high heterogeneity. HQT combined with mesalazine modulated the patients' serum IL-6, IL-10, IgA, and IgG levels. HQT combined with mesalazine for UC tended to reduce adverse effects; however, the difference was not statistically significant. All GRADE ratings of the quality of evidence were of low quality.

**Conclusions:**

HQT combined with mesalazine in the treatment of UC significantly improved the cure rate and overall treatment efficiency and regulated the expression levels of serum IL-6, IL-10, IgA, and IgG.

## 1. Introduction

Ulcerative colitis (UC) is a chronic nonspecific intestinal inflammatory disease characterized by continuous and diffuse inflammatory changes in the colorectal mucosa; however, its aetiology has not been fully understood. The lesions are mainly limited to the colorectal mucosa and the submucosa [1]. Clinical manifestations include recurrent diarrhea with mucus and pus, hematochezia, abdominal pain, and tenesmus with varying degrees of severity. It can also be accompanied by anemia, skin, and mucosal damage (such as oral ulcers and erythema nodosa), joint damage (such as peripheral or spinal arthritis), eye lesions (such as iritis or uveitis), metabolic bone disease, hepatobiliary system lesions (such as primary biliary cirrhosis PSC), and other extra-intestinal manifestations. The “Consensus Opinions on the Diagnosis and Treatment of Ulcerative Colitis with Integrated Traditional Chinese and Western Medicine 2017” proposes that the main points of UC diagnosis are typical clinical manifestations, endoscopic changes, and pathological diagnosis [1]. In 2019, the ACG Clinical Guideline: Ulcerative Colitis in Adults [2] pointed out that the assessment of disease severity is mainly used to guide treatment, and the assessment should be mainly based on (1) professional scale assessment (bleeding volume and stool frequency); (2) inflammation assessment (endoscopic assessment, including degree, severity, and markers of inflammation); (3) the course of disease (whether hospitalization is required and whether further treatment with hormones and other drugs may be required); and (4) impact of disease (physiological function and quality of life). The disease can occur at any age, and the peak incidence is mostly in young and middle-aged people aged 30–40, with no significant gender difference [3]. UC has now become a global disease and is most common in North America, Europe, and Australia. Several retrospective studies have shown that the incidence of UC is gradually stabilizing in Europe and the United States, while the incidence of UC is on the rise in non-Western countries, especially in Asia, South America, and eastern and southern Europe [4]. According to the aetiology, pathogenesis, and clinical manifestations of UC in traditional Chinese medicine, the disease is classified into the categories of “intestinal stagnation,” “diarrhoea,” “dysentery,” “intestinal wind,” and “dirty poison.” “Diarrhea” and “dysentery” are collectively referred to as “Xiali” [5].

Huangqin Tang (HQT) comes from Article 172 of the ShangHan Lun [6]. HQT is composed of four herbs: *Scutellaria baicalensis*, white peony root, liquorice root, and jujube. This prescription clears away heat, treats Xiali, and relieves pain. It is mainly used to treat abdominal pain and Xiali, which causes body heat and a bitter taste in the mouth, or dysentery and abdominal pain with heat, red tongue, and a stringy pulse [7]. In the prescription, the “king drug” *Scutellaria baicalensis* is bitter and cold, reduces turbidity, clears heat, and stops dysentery; the “official drug” *Chinese herbaceous peony* tastes sour, nourishes blood and astringes yin, and relieves pain; the auxiliary drugs liquorice and jujube relieve pain. The four herbs are used in combination for clearing heat, treating dysentery, and relieving urgency and pain. This formula is called “the ancestor of treating dysentery in all ages” in the Medical Prescriptions Collection as it forms the basis for many later classical prescriptions for dysentery treatment, such as baicalensis Shaoyao Tang for treating hot dysentery and abdominal pain and Shaoyao Tang for treating damp-heat dysentery. According to the latest clinical guidelines as well as consensus opinions [1, 2], mesalazine (5-aminosalicylic acid, 5-ASA) has been the first choice of treatment for mild to moderate UC. Several studies [8] have shown that 5-ASA induces endoscopic remission in moderate UC lesions to a degree similar to that of antitumor necrosis factor therapy. Bressler B [9] found that topical 5-ASA is superior to topical corticosteroids in inducing remission. Mesalazine has a favorable safety profile compared to immunomodulators and biologics. At present, HQT is widely used in the clinical treatment of UC, acute gastroenteritis, bacterial dysentery, and other diseases; however, there is no evidence-based medical basis for the treatment of UC by HQT combined with mesalazine. After reviewing a large number of research studies, our research group found that there was only a small amount of meta-analysis on the treatment of UC by HQT combined with sulphapyridine, and there was no systematic evaluation and meta-analysis on the evidence level of clinical studies on the treatment of UC by HQT combined with mesalazine. Earlier, our research group completed animal experiments on HQT combined with mesalazine for UC, and preliminary data indicated a significant curative effect. On this basis, we conducted a meta-analysis of HQT combined with mesalazine in the treatment of UC. This study aims to systematically evaluate the treatment of UC by HQT combined with mesalazine. The results of this study can provide a valuable reference for future clinical experiments and clinical applications of HQT in the treatment of UC.

## 2. Methods

### 2.1. Search Strategy and Study Selection

The CNKI, Wanfang Data, VIP, PubMed, SinoMed, Embase, and Cochrane Library databases were systematically searched from the establishment of each database to October 15, 2021. The Chinese database uses “Huangqin Tang” AND “ulcerative colitis” as the search mode, and supplementary search uses “Huangqin Tang,” “ulcerative colitis,” AND “inflammatory bowel disease” as the search terms and adopts the search mode of theme/keyword/abstract.

The English database search formula is (Huangqin Tang OR Huangqin Decoction OR Radix Scutellaria soup) AND (“nonspecific ulcerative colitis” OR “ulcerative Colitis” OR “ulcerative colitis” OR “ulcerous colitis” OR “colitis gravis”).

Subjects: we evaluated randomized controlled trials (RCTs) in which patients had a definitive diagnosis of ulcerative colitis; however, age, sex, and course of disease were not defined. There was no restriction on whether blinding was used in the study design. The intervention measures were HQT combined with mesalazine treatment and allowed for the addition of drugs in line with the requirements of the original prescription for the ShangHan Lun [6] based on the original prescription but excluding marked toxic drugs (refer to the 2020 edition of the People's Republic of China Pharmacopoeia [10]). The control drug mesalazine was recommended as the first-line drug in the clinical guidelines for ulcerative colitis [11], and the dosage form was not limited.

The main outcome indicators were cure rate and total effective rate. The secondary outcome measures were clinical symptom score (abdominal pain, diarrhea, hematochezia, and tenesmus) and levels of serum inflammatory factors including interleukin 6 (IL-6), interleukin 10 (IL-10), tumor necrosis factor *α* (TNF-*α*), serum immunoglobulin A (IgA), immunoglobulin M (IgM), and immunoglobulin G (IgG), and safety.

### 2.2. Data Extraction

Two researchers independently completed the literature retrieval through the search formula or search terms, screened out and excluded the literature that did not meet the inclusion criteria, and finally confirmed the literature selections. The third researcher compared the screening results. Any disagreements were resolved through discussion or by a third researcher. Two researchers independently extracted the data from the included literature and established the data extraction table: basic information, the methodological characteristics, the research object, intervention, outcome indicators, the results, and conclusions. Datasheets extracted by two researchers were compared, and a third researcher organized a discussion or resolution of different or divergent results.

### 2.3. Assessment of Methodological Quality

Referring to the Cochrane Handbook of Systematic Reviews [12], two researchers independently completed the quality assessment and bias risk assessment of the included studies using the risk of bias (ROB) tool in RevMan5.3, including the method of random sequence generation and hidden random-protocol allocation. They also noted if participants, people, and outcome assessments were blinded; if there was evidence of incomplete outcome data; and whether there was evidence of a risk of bias in the selective reporting of results. The evaluation results of the two researchers were compared, and a third researcher organized the discussion or resolution of the different or divergent results.

### 2.4. Statistical Analysis

The outcome index data of the included studies were entered into RevMan software (version 5.3). The relative risk (RR) meta-analysis was used for statistical analysis of the binary outcome index data, and the weighted mean difference (WMD) or standardized mean difference (SMD) meta-analysis was used for statistical analysis of the continuous outcome index data. The effect size was expressed with a 95% confidence interval (95% CI). The heterogeneity among the included studies was assessed. A fixed-effect model was adopted if the I2 between the results was less than 50%. If I^2^ was ≥50%, the random-effects model was adopted. Descriptive, systematic, or subgroup analyses were used if significant clinical heterogeneity existed between the included studies. The level of the meta-analysis was set at *α* = 0.05. The GRADE evidence quality grading system was used to evaluate the quality of evidence of the outcome indicators [13].

## 3. Results

### 3.1. Literature Search

A total of 411 original articles were retrieved from CNKI, Wanfang Data, VIP, PubMed, SinoMed, Embase, and the Cochrane Library. After preliminary screening, 225 articles were identified. In addition, 15 qualified articles were obtained through preliminary screening of literature titles and abstracts. After perusing the full text of the eligible literature, further screening was conducted according to the literature inclusion criteria. Finally, 6 studies were included, with a total of 565 patients.

### 3.2. Study Characteristics

A total of six studies were included [14–19], involving a total of 565 subjects with a definite diagnosis of UC, which were published in the last 5 years (2016–2021). The sample size of each study ranged from 68 to 126. The intervention was HQT plus mesalazine, and mesalazine was administered to the control group. The treatment course was 2 or 3 months, and the outcome indices included cure rate, effective rate, clinical symptom score, inflammatory factors, immunoglobulin levels, and adverse reactions. Further details are provided in Table 1.

### 3.3. Quality Assessment of the Included Studies

Among the six included studies, three used the random number table method to generate random sequences with a low risk of bias. The random sequence generation method of the remaining three studies was only described as “random” without specific explanation, indicating a high risk of bias. In blinding of outcome assessment, none of the six studies blinded the subjects, so the risk of bias could not be excluded. None of the six subjects dropped out; as a result, the risk of bias for incomplete outcomes was low. Moreover, none of the six studies mentioned whether the outcome evaluator was incomplete, and outcome bias was low. As it could not be determined whether the six study protocols were registered, the existence of reporting bias could not be ruled out (Figure 1).

### 3.4. Cure Rate and Total Efficiency Rate

Five studies that included cure rates [14–17, 19] were used to compare the difference in clinical cure rates between the HQT group and the control group—this included a total of 470 patients, with clinical heterogeneity I^2^ = 18%, <50%. Using the fixed-effect model, the meta-analysis results showed that the clinical cure rate of the HQT group was significantly higher than that of the control group (RR = 1.56, 95% CI (1.23, 1.98), *P*=0.0003) (see Figure 2(a)).

Five studies that included total efficiency rates [14–16, 16, 17] were used to compare the difference in clinical total efficiency rates between the HQT group and the control group. A total of 470 patients were included, with clinical heterogeneity I^2^ = 0%, <50%. Using the fixed-effect model, the meta-analysis results showed that the total clinical effective rate of the HQT group was significantly higher than that of the control group (RR = 1.24, 95% CI (1.14, 1.35), *P*=0.00001) (see Figure 2(b)).

### 3.5. Clinical Symptom Score

In total, 242 patients were included in the clinical symptom score study [14, 15]. The differences in the symptom scores of abdominal pain, diarrhea, hematochezia, and tenesmus were compared between the HQT and control groups. After careful reading of the literature scheme analysis, it was concluded that clinical heterogeneity I^2^ > 50% was caused by large differences in subjective scores. Using the random effect model, the meta-analysis results showed that the scores for diarrhea, hematochezia, and tenesmus in the HQT group were significantly lower than those in the control group, and there was no statistically significant difference in the scores for abdominal pain (diarrhea: SWD = −3.2, 95% CI (−5.81, −0.58), *P*=0.02; hematochezia: SWD = −4.12, 95% CI (−6.17, −2.08), *P*=0.00001; tenesmus: SWD = −3.14, 95% CI (−4.17, −2.12), *P*=0.00001; and abdominal pain: SWD = −2.97, 95% CI (−6.27, 0.33), *P* = 0.08).

### 3.6. Inflammatory Factors

Three studies included information on serum IL-10 levels [15, 18, 19], involving 289 patients. These studies were used to compare the differences in serum IL-10 levels between the HQT and control groups. Clinical heterogeneity I^2^ = 24%, <50%, fixed-effect model, and SMD meta-analysis results showed that HQT could significantly increase IL-10 content (SMD = 2.01, 95% CI (1.73, 2.30), *P*=0.00001) (see Figure 3(a)).

Two studies included serum IL-6 levels [15, 19], involving 194 patients. We used them to compare the difference in serum IL-6 levels between the HQT and control groups. Clinical heterogeneity I^2^ = 0%, <50%, fixed-effect model, and SMD meta-analysis results showed that HQT could significantly reduce IL-6 levels (SMD = −2.25, 95% CI (−2.61, −1.88), *P*=0.00001) (see Figure 3(b).

We analyzed three studies that included serum TNF-*α* levels [15, 18, 19], with a total of 289 patients, to compare the difference in serum TNF-*α* levels between the HQT and control groups. The clinical heterogeneity was I^2^ = 69%, >50%. This may be because the TNF-*α* data units in Yang M's experiment were different from those in the other two studies. The results of the meta-analysis using the random effect model and SMD showed that HQT could significantly reduce TNF-*α* levels (SMD = −1.45, 95% CI (−1.93, −0.97), *P*=0.00001).

### 3.7. Immunoglobulin

Two studies included immunoglobulin IgA [16, 18], involving 177 patients, with clinical heterogeneity of I^2^ = 0%, <50%. The fixed-effect model was adopted, and the results of the meta-analysis of SMD showed that the expression of immunoglobulin IgA in the HQT group was significantly decreased (SMD = −0.65, 95% CI (−0.96, −0.35), *P*=0.00001) (see Figure 4(a)).

Two studies included immunoglobulin IgM [16, 18], involving 177 patients, with clinical heterogeneity of I^2^ = 0% < 50%. The fixed-effect model was adopted, and the results of the meta-analysis of SMD showed that there was no significant difference in immunoglobulin IgM expression between the HQT and control groups (SMD = −0.09, 95% CI [−0.21, 0.38], *P*=0.56) (see Figure 4(b)).

Two studies included immunoglobulin IgG [16, 18], involving 177 patients, with clinical heterogeneity of I^2^ = 0%, <50%. The fixed-effect model was adopted, and the results of the meta-analysis of SMD showed that the expression level of immunoglobulin IgG in the HQT group was significantly decreased (SMD = −3.20, 95% CI (−3.65, −2.75), *P*=0.00001) (see Figure 4(c)).

### 3.8. Safety

Among the included studies, only one [17] reported safety. In the mesalazine group, eight patients showed adverse reactions, including 2 patients with nausea and vomiting, 3 patients with dizziness, and fatigue in 1 patient, and 2 patients with mild skin itching. In the HQT group, two patients showed adverse reactions, including one patient with nausea and vomiting and one patient with dizziness. We were able to contact the researchers of two studies [14, 15] by e-mail or telephone, and they replied that there were no adverse reactions. There was a trend of reduced adverse reactions in the adjuvant treatment of UC with HQT, but the difference was not statistically significant (RR = 0.25, 95% CI (0.06, 1.10), *P*=0.07).

### 3.9. Evaluation of GRADE Evidence Quality

The 13 outcome indicators were evaluated for evidence quality using GRADE. The evaluation results indicated the low quality of evidence. Further details are provided in Table 2.

## 4. Discussion

At present, the pathogenesis of UC has not been fully elucidated, but it is generally accepted that many factors, such as genetics, environment, and microorganisms, increase susceptibility to this disease. The resulting mucosal barrier changes, intestinal microflora disorders, and immune system defects cause sustained inflammatory reactions. One of the main pathogenic factors of UC is abnormal immune regulation. Both IL-6 and IL-10 play an important regulatory role in the development, differentiation, and immune response of immune cells; they participate in the activation of some cells and are closely related to the occurrence, development, and outcome of UC [20]. Western medicine treats UC by inhibiting intestinal inflammation. Commonly prescribed drugs for this illness include aminosalicylic acid, glucocorticoids, immunosuppressants, and biological agents, among which mesalazine and sulfasalazine are first-line drugs [2, 11]. The basic principles of traditional Chinese medicine in the treatment of UC are as follows: clearing heat and removing dampness; regulating qi and blood; astringing ulcers and promoting muscle during the active phase; strengthening the spleen and nourishing qi in the remission phase; supplementing the kidney and strengthening the root; and supplementing with clearing heat and removing dampness [21]. The pharmacodynamics studies showed that the main bioactive ingredients of HQT include baicalin, wogonoside, baicalein, wogonin and oroxylin-A, paeoniflorin, liquidity, and other herb components [22]. The main active ingredients of HQT for UC treatment are quercetin, kaempferol, baicalein, etc. [23–25]. The core targets are AKT1, JUN, IL6, VEGFA, STAT3, MYC, CASP3, EGFR, etc. [26]. The treatment of UC with HQT mainly acts on biological processes such as cancer pathway, MAPK signaling pathway, TNF signaling pathway, insulin resistance, JAK-STAT pathway, Th17 cell differentiation, NF-kB, and other signaling pathways, involving biological processes such as endotoxin response, regulation of apoptosis signaling pathway, regulation of small molecule metabolic process, reactive oxygen metabolic process, and negative regulation of cell proliferation [27]. Besides, some existing basic studies have shown that HQT may play a role in the treatment of UC through multiple targets and mechanisms; for example, by inhibiting the activation of IL-6, JAK, and STAT3 signaling pathways and the expression of HGBB-1, it can reduce the production of inflammatory cytokines and inflammatory responses, thus improving intestinal function and restoring intestinal structure [28]. The intestinal immune system is regulated by the expression of various cytokines, such as IL-6, IL1-*β*, and IL-10, to maintain homeostasis of the intestinal mucosal system [26]. By promoting the expression of the MHC II molecule and increasing ILC3 s cells, upregulating the expression of Treg cells and downregulating the expression of Th1 cells, inhibiting the secretion of a variety of proinflammatory factors, and then regulating the immune response of Th cells, DSS-induced mouse ulcerative colitis is alleviated [29].

Multicentre, large-sample RCTs have achieved the highest level of evidence-based medical evidence [30]. In recent years, the number of RCT studies on the treatment of UC by HQT has increased significantly. However, there is no systematic evaluation of the level of evidence in clinical studies of HQT combined with mesalazine for the treatment of UC. Six studies were included in this meta-analysis, and the results showed that HQT combined with mesalazine in the treatment of UC could significantly improve the cure rate and total effective rate, as well as the expression levels of IL-6, IL-10, IgA, and IgG in the serum of patients. However, there was no statistical difference in the expression of serum IgM. Clinical symptom scores have high heterogeneity, which may be caused by large differences in subjective scores. Heterogeneity was also high in the meta-analysis of the effects on TNF-*α*, which may be because the data unit of TNF-*α* in Yang's experiment was different from that in the other two studies. Few reports provide data on adverse reactions; the effect of HQT on reducing the incidence of adverse reactions thus still needs to be verified by further studies. The limitations of this meta-analysis are as follows: (1) The sample size was small, and the experimental studies investigated were not rigorously designed. Among the included studies, only three described the random number table method for random sampling and none of them mentioned whether the blind method was adopted or whether allocation hiding was set, which has a high risk of bias. (2) Most of the articles only evaluated the efficacy rate, cure rate, and clinical symptoms; the clinical symptom score standard was not uniform and highly subjective, leading to high heterogeneity. (3) There was a lack of evaluation studies using objective indicators, such as the efficacy of colonoscopy and mucosal histology, and the data units of test indicators were inconsistent in some studies. (4) There was a lack of detailed reports on adverse reactions; furthermore, it was difficult to obtain contact details that could be accessed to obtain further information. (5) The course of HQT combined with mesalazine in the treatment of UC is not clear, and regular follow-up or follow-up results have not been reported.

Therefore, the results of this study suggest that the following aspects should be emphasized in later clinical trials of HQT for UC: (1) Expand the sample size, design a more scientific and rigorous randomized controlled trial, reduce risk bias as much as possible, improve the methodological quality, adopt standardized randomized methods, and allocate hidden and blind methods. (2) Strengthen the evaluation of clinical symptoms, colonoscopic efficacy, and mucosal histology and recommend the use of unified scoring criteria, such as the Modified Mayo Disease Activity Index and Original Geboes Score. (3) For the determination of serum or colon markers, high-quality immunokits should be used as far as possible, and strictly standardized operations should be performed. Possible detection indexes include serum IL-6, IL-1*β*, IL-10, TNF-*α*, COX2, routine blood examination, routine fecal examination, plasma protein, ESR, CRP, and fecal calprotectin (4) Gather detailed data on adverse reactions and the safety of TCM compounds. (5) Gather data on the patients' quality of life, evaluate the patient's psychological and mental state, stage follow-up, and make detailed reports in the literature.

## 5. Conclusions

HQT combined with mesalazine in the treatment of UC significantly improved the cure rate and overall treatment efficiency and regulated the expression levels of serum IL-6, IL-10, IgA, and IgG.

## Figures and Tables

**Figure 1:** Included study bias risk assessment.

**Figure 2:** Meta-analysis of cure rate (a) and total efficiency (b) of the HQT group compared with the mesalazine group.

**Figure 3:** Meta-analysis of IL-10 (a) and IL-6 (b) content in the HQT group compared with the mesalazine group.

**Figure 4:** Meta-analysis of IgA (a) IgM (b) and IgG (c) content in the HQT group compared with the mesalazine group.

**Table 1:** Characteristics of the included literature.

Author, year	Sample size	Diagnostic criteria	Male%	Age (years)		Course of the disease		Treatment intervention	Control intervention	Period of treatment (months)	Outcome indicator
				Experimental group	Control group	Experimental group	Control group				
Hu et al., [14]	116	Clinical symptoms, colonoscopy, pathology	51.7%	42.37 ± 2.87	42.61 ± 2.82	8.71 ± 2.42	8.94 ± 2.4	HQT^1^+mesalazine^a^	Mesalazine^a^	2	Cure rate, total effective rate, clinical symptom score
Ding et al., [15]	126	Clinical symptoms, colonoscopy, pathology	53.2%	43.5 ± 9.6	42.4 ± 8.7	9.5 ± 3.2	9.2 ± 3.5	HQT^2^+mesalazine^a^	Mesalazine^a^	2	Cure rate, total effective rate, TCM syndrome score, IL-6/10/TNF-*α* IgG/IgM/IgA
Yan [16]	82	Clinical symptoms, imaging	54.9%	36.68 ± 6.52	36.74 ± 6.58	6.52 ± 3.23	6.47 ± 3.18	HQT^1^+mesalazine^a^	Mesalazine^a^	2	Cure rate, total effective rate
Wang and Wang [17]	78	Clinical symptoms, colonoscopy	57.7%	35.36 ± 4.32	35.18 ± 4.29	3.91 ± 0.45	3.86 ± 0.41	HQT^1^+mesalazine	Mesalazine	3	Cure rate, total effective rate, adverse reactions
Lu [18]	95	Clinical symptoms, colonoscopy, pathology	51.6%	36.57 ± 6.59	35.97 ± 6.29	NA	NA	HQT^1^+mesalazine^b^	Mesalazine^b^	2	IL-10/TNF-*α*,IgG/IgM/IgA
Yang [19]	68	Clinical symptoms, colonoscopy, pathology, imaging	48.5	42.6 ± 12.7	41.5 ± 12.5	NA	NA	HQT^2^+mesalazine^b^	Mesalazine^b^	2	Cure rate, total effective rate, IL-6/10/TNF-*α*

“1” represents decoction of HQT, “2” represents granule of HQT; “a” represents mesalazine granules or sustained-release granules, and “b” represents mesalazine enteric-coated tablets.

**Table 2:** GRADE summary of HQT in the UC randomized controlled trial.

			Evaluation of evidence quality					
Outcome	Number of studies	Study design	Risk of bias	Inconsistency	Indirectness	Imprecision	Quality (evidence)	Importance of outcome
Cure rate	5	RCT	Serious^a^	Serious^b^	Not serious	Not serious	Low	Critical
Total effective rate	5	RCT	Serious^a^	Not serious	Not serious	Not serious	Low	Critical
Diarrhea	2	RCT	Serious^c^	Serious^d^	Not serious	Not serious^gh^	Low	Important
Abdominal pain	2	RCT	Serious^b^	Serious^d^	Not serious	Not serious^gh^	Low	Important
Hematochezia	2	RCT	Serious^b^	Serious^d^	Not serious	Serious^gh^	Low	Important
Tenesmus	2	RCT	Serious^b^	Serious^d^	Not serious	Serious^gh^	Low	Important
TNF-*α*	3	RCT	Serious^e^	Serious^f^	Not serious	Not serious	Low	Important
IL-10	3	RCT	Serious^e^	Not serious	Not serious	Not serious	Low	Important
IL-6	2	RCT	Serious^c^	Not serious	Not serious	Serious^gh^	Low	Important
IgM	2	RCT	Serious^c^	Not serious	Not serious	Serious^gh^	Low	Not important
IgG	2	RCT	Serious^c^	Not serious	Not serious	Serious^gh^	Low	Not important
IgA	2	RCT	Serious^c^	Not serious	Not serious	Serious^gh^	Low	Not important
Safety	3	RCT	Serious^e^	Not serious	Not serious	Not serious	Low	Important

^a^Three studies used the random number table method; it was unclear whether the blind method was used, and random conceals were not reported. ^b^One study used a significant effect description in which the requirements for clinical symptoms and colonoscopy observation met the cure criteria. ^c^One study used the random number table method; it was unclear whether the blind method was used, and random conceals were not reported. ^d^There are operational differences in the clinical symptom score rules. ^e^Two studies adopted the random number table method, but it was not clear whether the blind method was adopted. ^f^The experimental data units of one study differed from those of the other studies. ^g^Small sample size. ^h^Low event rate.

## Data Availability

The datasets presented in this study can be found in the online repositories. System evaluation registration: International Prospective System Evaluation Registration Platform (PROSPERO), CRD42021234614.
